This article has been retracted.

# Evaluate teaching quality of physical education using a hybrid multi-criteria decision-making framework

**DOI:** 10.1371/journal.pone.0280845

**Published:** 2023-02-16

**Authors:** Zhenyin Chen, Suizhi Luo

**Affiliations:** 1 Sports Department of Physical Education, Central South University, Changsha, China; 2 College of Tourism, Hunan Normal University, Changsha, China; University of Belgrade Faculty of Organisational Sciences: Univerzitet u Beogradu Fakultet organizacionih nauka, SERBIA

## Abstract

The teaching quality evaluation of physical education is an important measure to promote the professional development of physical teachers, improve the quality of school teaching and personnel training. It is helpful for students to achieve all-round development and better meet the needs of modern talents in the new era. This study aims to establish a novel MCDM (multi-criteria decision-making) framework for evaluating teaching quality of physical education. First, PFNs (picture fuzzy numbers) are suggested to reflect dissimilar attitudes or preferences of decision makers. Then, the typical SWARA (Step-wise Weight Assessment Ratio Analysis) model is modified with PFNs to calculate the weights of evaluation criteria. Considering that some criteria are non-compensatory during the evaluation process, the idea of ELECTRE (elimination and choice translating reality) is introduced to obtain the ranking results of alternatives. Specially, the MAIRCA (Multi-Attribute Ideal-Real Comparative Analysis) method is extended to construct the difference matrix in a picture fuzzy environment. Last, the hybrid MCDM model is utilized to assess the teaching quality of physical education. Its superiority is justified through comparison analyses. Results show that our approach is practicable and can provide instructions for the teaching quality evaluation of physical education.

## Introduction

As a key component of school education, school physical education plays a vital role in promoting students’ all-round development and cultivating students’ innovative spirit and practical ability [1]. The teaching quality evaluation of physical education can not only effectively control the implementation and reform of physical education teaching, but also be used in the training, recruitment and selection of physical education teachers [2]. Scientific teaching quality evaluation system and methods are very important to improve the quality of school teaching and train sports professionals. Some researchers have focused on the teaching quality evaluation of physical education. Recently, Zeng [3] evaluated physical education teaching quality based on the data mining technology and hidden Markov model; Duan and Hou [4] solved the teaching quality evaluation problems with the simulated annealing algorithm; Cheng [5] introduced web embedded system and virtual reality to assess teaching quality of physical education; Williams et al. [6] discussed the teach quality of physical education using psychology, a Game Sense Approach and the Aboriginal game Buroinjin. However, these methods are qualitative or applied only to certain decision-making environments.

Jiang and Wang [7] established a fuzzy comprehensive evaluation model for evaluating teaching quality of public physical education; Mishra et al. [8] assessed physical education teaching quality based on intuitionistic fuzzy similarity measures; Liu [9] established an intuitionistic fuzzy TOPSIS (Technique for Order Preference by Similarity to an Ideal Solution) model for the teaching quality evaluation of physical education. To evaluate the teaching quality of physical education more comprehensively, evaluators from many sides, such as field experts, authorities and students, are usually needed. In such a case, multiple dissimilar attitudes or perceptions may arise at the same time. Therefore, PFNs (picture fuzzy numbers) [10] are suggested to describe uncertain evaluation information. The most obvious feature of PFNs is it that it contains four different membership functions, which can accommodate diverse viewpoints and describe decision makers’ ambiguity, uncertainty and inconsistency sufficiently.

To date, plenty of decision-making methods have been extended for tackling evaluation issues under picture fuzzy circumstances [11]. Some researchers established various picture fuzzy decision-making models based on dissimilar aggregation operators. For example, Wei [12] defined the arithmetic and geometric aggregation operators with picture fuzzy information; Khan et al. [13] discussed the picture fuzzy Logarithmic aggregation operators; Jana et al. [14] introduced the picture fuzzy Dombi aggregation operators; Ateş and Akay [15] extended the Bonferroni mean operators in picture fuzzy environments; Jin et al. [16] explored the weighted interaction arithmetic and geometric aggregation operators with PFNs; and Ashraf et al. [17] proposed some Maclaurin symmetric mean operators in picture fuzzy environments. However, they may lead to information loss or distortion during the aggregation process.

Liang et al. [18] integrated the EDAS (evaluation based on the distance from average solution) with ELECTRE (elimination and choice translating reality) models for evaluating cleaner production of mines; Wang et al. [19] investigated the picture fuzzy MABAC (multi-attributive border approximation area comparison) technique to solve risk assessment problems of energy contracting projects; Ashraf et al. [20] modified the TOPSIS method for solving decision-making issues in picture fuzzy surroundings; Wei et al. [21] presented a picture fuzzy bidirectional projection approach to assess safety of construction project; Luo et al. [22] selected the site of tailings pond with an extended WDBA (Weighted Distance Based Approximation) method under picture fuzzy circumstances; Gündoğdu et al. [23] assessed public transport service quality with the AHP (Analytic Hierarchy Process) and linear assignment model in picture fuzzy surroundings; Aydoğmuş et al. [24] developed a CODAS (Combinative Distance-based Assessment) algorithm to select suitable ERP (Enterprise Resource Planning) systems within picture fuzzy situations; Korucuk et al. [25] proposed a CoCoSo (combined compromise solution) method with PFNs for evaluating ideal smart network strategies for logistics companies; Gireesha et al. [26] introduced a picture fuzzy MARCOS (Measurement of Alternatives and Ranking according to Compromise Solution) method to assess could service; and Yildirim and Yıldırım [27] modified VIKOR (VlseKriterijuska Optimizacija I Komoromisno Resenje) approach with picture fuzzy information to assess the satisfaction level of citizens in municipality services.

Recently, a novel multi-criteria evaluation method, the MAIRCA (Multi-Attribute Ideal-Real Comparative Analysis), was proposed by Pamucar et al. [28]. It obtains the ranking orders of alternatives based on the gap between theoretical and real results [29]. Nevertheless, the classical MAIRCA approach with exact numbers cannot capture decision makers’ ambiguity and vagueness. In this case, few scholars combined MAIRCA with fuzzy set theory to resolve decision-making issues. For instances, Chatterjee et al. [30] Evaluated the performance of suppliers with a rough MAIRCA technique for green supply chain implementation in electronics industry; Adar and Kilic Delice [31] modified the MAIRCA model with hesitant fuzzy linguistic term sets; Boral et al. [32] integrated AHP with MAIRCA in a fuzzy environment for fuzzy failure modes and effects analysis; Bagheri et al. [33] identified the uncertainty factors on the constructional project with an extended MAIRCA under hesitant fuzzy circumstances; García Mestanza and Bakhat [34] presented a fuzzy MAIRCA for evaluating over-tourism; Zhu et al. [35] established an extended MAIRCA model to assess biological inspiration for biologically inspired design in fuzzy rough environments; Ecer [36] modified the MAIRCA with intuitionistic fuzzy numbers to choose coronavirus vaccine in the age of COVID-19. However, the MAIRCA has neither been extended in a picture fuzzy environment, nor been utilized to deal with teaching quality evaluation issues.

In view of the above inspiration, the intention of this study is to investigate the physical education teaching quality evaluation problem under a picture fuzzy environment, which has strong theoretical and practical significance. The major innovation and contribution are: First, PFNs are utilized to depict complex and fuzzy evaluation information. As a result, different opinions and judgments of decision makers can be expressed with four membership functions. Second, the classical SWARA (Step-wise Weight Assessment Ratio Analysis) is extended with PFNs to compute criteria weights. Third, a new MCDM (multi-criteria decision-making) method is proposed. In this framework, the idea of MAIRCA is introduced to construct difference matrix, while the ELECTRE method is modified to obtain ranking results in picture fuzzy environment. Fourth, the hybrid MAIRCA-ELECTRE method is utilized to tackle teaching quality evaluation problems of physical education. Further, its feasibility and effectiveness are proved.

The rest is outlined as follows. Preliminaries of PFS and PFNs are described in Section 2; a new methodology, the hybrid MAIRCA-ELECTRE method, is developed with four phases in Section 3; a case of teaching quality evaluation of physical education is studied to testify the feasibility of our approach in Section 4; comparison analyses and discussions are made to verify the efficiency of the MAIRCA-ELECTRE method in Section 5; and final conclusions are drawn in Section 6.

### Preliminaries

#### Definition 1

[10] Given three membership degrees *a*(*θ*), *b*(*θ*) and *c*(*θ*), then *α*(*θ*) = {< *θ*, *a*(*θ*), *b*(*θ*), *c*(*θ*) > |*θ* ∈ *Ω*} is a PFS (picture fuzzy set) on a universe Ω, where 0 ≤ *a*(*θ*) ≤ 1, 0 ≤ *b*(*θ*) ≤ 1, 0 ≤ *c*(*θ*) ≤ 1 and 0 ≤ *e*(*θ*) = 1—*a*(*θ*)- *b*(*θ*)—*c*(*θ*) ≤ 1 is the positive, neutral, negative and refusal membership degree, respectively.

Specifically, when only one element exists in a PFS, it is degraded into a PFN (picture fuzzy number) *α* = (*a*, *b*, *c*).

#### Definition 2

[10] For two PFNs *α*_1_ = (*a*_1_, *b*_1_, *c*_1_) and *α*_2_ = (*a*_2_, *b*_2_, *c*_2_), their operational rules include

1. $\alpha_{1}⊕\alpha_{2}=(a_{1}+a_{2}-a_{1}a_{2},b_{1}b_{2},c_{1}c_{2})$;
2. $\alpha_{1}⊗\alpha_{2}=(a_{1}a_{2},b_{1}+b_{2}-b_{1}b_{2},c_{1}+c_{2}-c_{1}c_{2})$;
3. $\vartheta \cdot \alpha_{1}=(1-{\left(1-a_{1}\right)}^{\vartheta },b_{1}{}^{\vartheta },c_{1}{}^{\vartheta })$ (ϑ>0);
4. $\alpha_{1}{}^{\vartheta }=(a_{1}{}^{\vartheta },1-{\left(1-b_{1}\right)}^{\vartheta },1-{\left(1-c_{1}\right)}^{\vartheta })$ (ϑ>0).

#### Definition 3

[11] If *α* = (*a*, *b*, *c*) is a PFN, its score function *S*(*α*) can be defined as

S(α)=a−c, (1)

#### Definition 4

[11] If *α* = (*a*, *b*, *c*) is a PFN, its accuracy function *A*(*α*) can be defined as

A(α)=a+b+c. (2)

#### Definition 5

[18] Assume *α*_1_ = (*a*_1_, *b*_1_, *c*_1_) and *α*_2_ = (*a*_2_, *b*_2_, *c*_2_) are two arbitrary PFNs, then

1. $\alpha_{1}≻\alpha_{2}$ if $\left\{\begin{array}{c} S(\alpha_{1})>S(\alpha_{2})\\ S(\alpha_{1})=S(\alpha_{2})\;and\;A(\alpha_{1})>A(\alpha_{2})\; \end{array}\right.$;
2. $\alpha_{1}≺\alpha_{2}$ if $\left\{\begin{array}{c} S(\alpha_{1})<S(\alpha_{2})\\ S(\alpha_{1})=S(\alpha_{2})\;and\;A(\alpha_{1})<A(\alpha_{2}) \end{array}\right.$;
3. $\alpha_{1}∼\alpha_{2}$ if $S(\alpha_{1})=S(\alpha_{2})$ and $A(\alpha_{1})=A(\alpha_{2})$.

#### Definition 6

[18] If *α*_1_ = (*a*_1_, *b*_1_, *c*_1_) and *α*_2_ = (*a*_2_, *b*_2_, *c*_2_) are two arbitrary PFNs, then their Euclidean distance is

$$d(\alpha_{1},\alpha_{2})=\sqrt{\left(|a_{1}-a_{2}{|}^{2}+|b_{1}-b_{2}{|}^{2}+|c_{1}-c_{2}{|}^{2}+|e_{1}-e_{2}{|}^{2}\right)}.$$ (3)

## Hybrid multi-criteria decision-making framework

In this section, a hybrid decision-making framework is established to deal with multi-criteria evaluation issues in picture fuzzy environments. The flowchart of this method is shown in **Fig 1**.

**Fig 1:** Flowchart of the proposed methodology.

### Phase I: Establishment of assessment matrix

In this phase, decision-making information is acquired under picture fuzzy circumstances. Afterwards, a standard assessment matrix is constructed by normalizing the original evaluation data.

**Step 1:** Attain initial evaluation data.

Considering decision-making issues with some alternatives {*A*_1_, *A*_2_,…, *A*_*m*_} in picture fuzzy environments, experts first determine the evaluation criteria {*C*_1_, *C*_2_,…, *C*_*n*_} and their corresponding weights (*ω*_1_, *ω*_2_,…, *ω*_*n*_), where *ω*_*j*_ ∈ [0,1] and $\sum_{j=1}^{n}\omega_{j}=1$. Thereafter, they try to assess each alternatives under these criteria and construct an evaluation matrix $E={\left(\alpha_{ij}\right)}_{m\times n}=\begin{array}{cc} & \begin{array}{cccc} C_{1} & C_{2} & \cdots & C_{n} \end{array}\\ \begin{array}{c} A_{1}\\ A_{2}\\ \vdots \\ A_{m} \end{array} & \left[\begin{array}{cccc} \alpha_{11} & \alpha_{12} & \cdots & \alpha_{1n}\\ \alpha_{21} & \alpha_{22} & \cdots & \alpha_{2n}\\ \vdots & \vdots & & \vdots \\ \alpha_{m1} & \alpha_{m2} & \cdots & \alpha_{mn} \end{array}\right] \end{array}$ where *α*_*ij*_ = (*a*_*ij*_, *b*_*ij*_, *c*_*ij*_) (*i* = 1, 2,…, *m*; *j* = 1, 2,…, *n*) is a PFN.

**Step 2:** Normalize the initial decision-making matrix.

When evaluation criteria belong to different types (benefit or cost criteria), they need to be normalized with

$${\tilde{\alpha }}_{ij}=({\tilde{a}}_{ij},{\tilde{b}}_{ij},{\tilde{c}}_{ij})=\left\{\begin{array}{c} (a_{ij},b_{ij},c_{ij})\;for\;benefit\;criteria\\ (c_{ij},b_{ij},a_{ij})\;for\;\cos t\;criteria \end{array}\right..$$ (4)

Consequently, a normalized decision-matrix $\tilde{E}={\left({\tilde{\alpha }}_{ij}\right)}_{m\times n}$ can be established.

### Phase II: Determination of criteria weights using modified SWARA method

In this phase, the criteria weight values are calculated using a modified SWARA method under picture fuzzy contexts.

**Step 1:** Get a descending order of criteria.

Decision makers rank all evaluation criteria according to the significance of criteria, their knowledge, experience and preference. The most important criterion comes first, followed by the less important criterion, until a descending order of criteria *C*_(1)_ ≻ *C*_(2)_≻…≻ *C*_(*n*)_ is obtained.

**Step 2:** Compute the comparative importance index.

Experts are asked to estimate the comparative importance degree of criterion *C*_(*j*-1)_ over *C*_(*j*)_ with a PFN *β*_*j*_ = (*a*_*j*_, *b*_*j*_, *c*_*j*_) (*a*_*j*_ ≥ 0.5), then the comparative importance index *p*_(*j*)_ can be computed with

$$p_{\left(j\right)}=S(\beta_{j})(j=2,3,\ldots ,n).$$ (5)

**Step 3:** Calculate the importance degree of each criterion.

According to the comparative importance index, the importance degree is

$$r_{\left(j\right)}=\left\{\begin{array}{c} 1,\;j=1\\ r_{\left(j-1\right)}/(p_{\left(j\right)}+1),\;j=2,3,\ldots ,n \end{array}\right..$$ (6)

**Step 4:** Obtain the weight values of criteria.

The criteria weights can be obtained with

$$\omega_{\left(j\right)}=r_{\left(j\right)}/\sum_{j=1}^{n}r_{\left(j\right)},\;(j=1,2,\ldots ,n).$$ (7)

### Phase III: Construction of difference matrix using extended MAIRCA approach

In this phase, the idea of MAIRCA method is borrowed to construct a difference matrix.

**Step 1:** Obtain the picture fuzzy priority for the selection of each alternative.

Generally, experts are unbiased with each alternative before making decisions. That is, they have no preference for any certain alternative. In this case, the picture fuzzy priority $P_{A_{i}}$ (*i* = 1,2,…, *m*) for the selection of each alternative is visually equivalent, denoted as

$$P_{A_{1}}=P_{A_{2}}=\cdots =P_{A_{m}}=\frac{1}{m}.$$ (8)

**Step 2:** Establish the theoretical assessment matrix.

According to [28], the elements in a theoretical assessment matrix are the coefficient of the preference picture fuzzy priority $P_{A_{1}}$ (*i* = 1,2,…, *m*) and the criteria weight *ω*_*j*_ (*j* = 1,2,…, *n*), namely, $t_{ij}=P_{A_{i}}\cdot \omega_{j}$. Therefore, a *m* × *n* theoretical assessment matrix *T* can be established as follows:

$$T={\left(t_{ij}\right)}_{m\times n}=\begin{array}{cc} & \begin{array}{cccc} \omega_{1} & \omega_{2} & \cdots & \omega_{n} \end{array}\\ \begin{array}{c} P_{A_{1}}\\ P_{A_{2}}\\ \vdots \\ P_{A_{m}} \end{array} & \left[\begin{array}{cccc} t_{11} & t_{12} & \cdots & t_{1n}\\ t_{21} & t_{22} & \cdots & t_{2n}\\ \vdots & \vdots & & \vdots \\ t_{m1} & t_{m2} & \cdots & t_{mn} \end{array}\right] \end{array}=\begin{array}{cc} & \begin{array}{cccc} \omega_{1} & \omega_{2} & \cdots & \omega_{n} \end{array}\\ \begin{array}{c} P_{A_{1}}\\ P_{A_{2}}\\ \vdots \\ P_{A_{m}} \end{array} & \left[\begin{array}{cccc} P_{A_{1}}\omega_{1} & P_{A_{1}}\omega_{2} & \cdots & P_{A_{1}}\omega_{n}\\ P_{A_{2}}\omega_{1} & P_{A_{2}}\omega_{2} & \cdots & P_{A_{2}}\omega_{n}\\ \vdots & \vdots & & \vdots \\ P_{A_{m}}\omega_{1} & P_{A_{m}}\omega_{2} & \cdots & P_{A_{m}}\omega_{n} \end{array}\right] \end{array}.$$ (9)

**Step 3:** Establish the real assessment matrix.

Based on the initial normalized evaluation matrix and the theoretical assessment matrix, a real assessment matrix *R* can be established as follows:

$$R={\left(r_{ij}\right)}_{m\times n}=\begin{array}{cc} & \begin{array}{cccc} C_{1} & C_{2} & \cdots & C_{n} \end{array}\\ \begin{array}{c} A_{1}\\ A_{2}\\ \vdots \\ A_{m} \end{array} & \left[\begin{array}{cccc} r_{11} & r_{12} & \cdots & r_{1n}\\ r_{21} & r_{22} & \cdots & r_{2n}\\ \vdots & \vdots & & \vdots \\ r_{m1} & r_{m2} & \cdots & r_{mn} \end{array}\right] \end{array},$$ (10)

where $r_{ij}=t_{ij}\cdot \frac{d({\tilde{\alpha }}_{ij},{\tilde{\alpha }}_{j}^{-})}{d({\tilde{\alpha }}_{j}^{+},{\tilde{\alpha }}_{j}^{-})}$, $d({\tilde{\alpha }}_{ij},{\tilde{\alpha }}_{j}^{-})$ is the distance between ${\tilde{\alpha }}_{ij}$ and ${\tilde{\alpha }}_{j}^{-}$, $d({\tilde{\alpha }}_{j}^{+},{\tilde{\alpha }}_{j}^{-})$ is the distance between ${\tilde{\alpha }}_{j}^{+}$ and ${\tilde{\alpha }}_{j}^{-}$, ${\tilde{\alpha }}_{j}^{-}=\min({\tilde{\alpha }}_{1j},{\tilde{\alpha }}_{2j},\cdots ,{\tilde{\alpha }}_{mj})$ is the minimum value of alternatives under criterion *C*_*j*_, ${\tilde{\alpha }}_{j}^{+}=\max({\tilde{\alpha }}_{1j},{\tilde{\alpha }}_{2j},\cdots ,{\tilde{\alpha }}_{mj})$ is the maximum value of alternatives under criterion *C*_*j*_, and ${\tilde{\alpha }}_{ij}$ is initial normalized evaluation value, denoted as a PFN.

**Step 4:** Construct the difference matrix.

Based on the theoretical and the real assessment matrices, their gap can be formed into a difference matrix *G* as follows:

$$G=T-R={\left(g_{ij}\right)}_{m\times n}=\left[\begin{array}{cccc} g_{11} & g_{12} & \cdots & g_{1n}\\ g_{21} & g_{22} & \cdots & g_{2n}\\ \vdots & \vdots & & \vdots \\ g_{m1} & g_{m2} & \cdots & g_{mn} \end{array}\right]=\left[\begin{array}{cccc} t_{11}-r_{11} & t_{12}-r_{12} & \cdots & t_{1n}-r_{1n}\\ t_{21}-r_{21} & t_{22}-r_{22} & \cdots & t_{2n}-r_{2n}\\ \vdots & \vdots & & \vdots \\ t_{m1}-r_{m1} & t_{m2}-r_{m2} & \cdots & t_{mn}-r_{mn} \end{array}\right].$$ (11)

### Phase IV: Acquisition of ranking orders using ELECTRE III method

In this phase, the ELECTRE III method is adopted for obtaining the alternatives’ ranks.

**Step 1:** Calculate the concordance degree between two alternatives.

The concordance degree between *A*_*i*_ and *A*_*k*_ (*i*, *k* = 1,2,…, *m*) can be calculated with

$$CD(A_{i},A_{k})=\sum_{j=1}^{m}\left(\omega_{j}\cdot \Psi (g_{ij},g_{kj})\right),$$ (12)

where $\Psi (g_{ij},g_{kj})=\left\{\begin{array}{c} \;1,\;g_{ij}-g_{kj}\leq \nabla_{j}\;\\ \frac{\Delta_{j}-(g_{ij}-g_{kj})}{\Delta_{j}-\nabla_{j}},\;\nabla_{j}<g_{ij}-g_{kj}<\Delta_{j}\\ 0,\;g_{ij}-g_{kj}\geq \Delta_{j} \end{array}\right.$, ∇_j_ and Δ_*j*_ are the preference and indifference thresholds under criterion *C*_*j*_, and 0 ≤ ∇_*j*_ < *j*.

**Step 2:** Compute the credibility degree between two alternatives.

The credibility degree between *A*_*i*_ and *A*_*k*_ (*i*,*k* = 1,2,…,*m*) can be calculated with

$$CI(A_{i},A_{k})=CD(A_{i},A_{k})\cdot \prod_{j=1}^{m}DI_{j}(A_{i},A_{k}),$$ (13)

where $DI_{j}(A_{i},A_{k})=\left\{\begin{array}{c} \;1,\;ϒ(g_{ij},g_{kj})\leq CD(A_{i},A_{k})\\ \;\frac{1-ϒ(g_{ij},g_{kj})}{1-CD(A_{i},A_{k})},\;ϒ(g_{ij},g_{kj})>CD(A_{i},A_{k}) \end{array}\right.$, $ϒ(g_{ij},g_{kj})=\left\{\begin{array}{c} 1,\;g_{ij}-g_{kj}\geq \Lambda_{j}\\ \frac{g_{ij}-g_{kj}-\Delta_{j}}{\Lambda_{j}-\Delta_{j}},\;\Delta_{j}<g_{ij}-g_{kj}<\Lambda_{j}\\ \;0,\;g_{ij}-g_{kj}\leq \Delta_{j}\; \end{array}\right.$ and 0 ≤ *Δ*_*j*_ < *Λ*_*j*_.

**Step 3:** Acquire the ranks according to the ranking index.

The ranking index of *A*_*i*_(*i* = 1,2,…,*n*) can be determined by

$$RI(A_{i})=\sum_{k=1}^{n}CI(A_{i},A_{k})-\sum_{k=1}^{n}CI(A_{k},A_{i}).$$ (14)

As a result, the alternatives’ ranks are acquired based on the values of *RI*(*A*_*i*_). Namely, the bigger the value of *RI*(*A*_*i*_), the better the alternative *A*_*i*_, and the best alternative A* has the biggest value of *RI*(A*) = *max*(*RI*(*A*_*i*_)).

## Case study

In this section, a case of teaching quality evaluation of physical education is investigated.

### Background

Physical education is an indispensable part of the development of education. It aims to cultivate more excellent comprehensive talents for the country and is an important cornerstone to promote the vigorous development of various undertakings. The teaching quality evaluation criteria system of physical education is shown in **Table 1** [4].

**Table 1:** Teaching quality evaluation criteria system of physical education [4].

Criterion	Type	Description
Teaching attitude *C*_1_	Benefit	It is mainly reflected by teaching style, teaching discipline, class spirit, teachers’ sense of responsibility and initiative.
Teaching contents *C*_2_	Benefit	It is mainly reflected by the amount of information, key points, appropriateness and advancement of contents.
Teaching approaches *C*_3_	Benefit	It is mainly reflected by effective organization, active classroom atmosphere, and students’ mobilized enthusiasm.
Teaching effect *C*_4_	Benefit	It is mainly reflected by teachers’ clear explanations, useful extracurricular homework, and developments of students’ ability.
Teaching link *C*_5_	Benefit	It is mainly reflected by adequate lesson preparation, quality of extracurricular training homework and use of advanced teaching technology.

### Illustration

Suppose there are four physical education colleges {*A*_1_, *A*_2_, *A*_3_, *A*_4_}, the proposed methodology in Section 4 is adopted to evaluate their teaching quality.

In Phase I, the assessment matrix is constructed in a picture fuzzy context. First, ten decision makers (including four government representatives related to physical education, four professionals and scholars in the field of physical education, and two sports practitioners) are organized to make assessments for them based on **Table 1**. In view of the unquantifiable nature of most criteria, PFNs are finally used to describe the evaluation results. As a result, an initial decision-making matrix can be built, as shown in **Table 2**. Because five evaluation criteria are all benefit criteria, they do not need to be normalized. Namely, the normalized decision-making matrix is the same as the initial matrix.

**Table 2:** Initial evaluation matrix *E*.

*E*	*C*_1_	*C*_2_	*C*_3_	*C*_4_	*C*_5_
*A*_1_	(0.7,0.2,0.1)	(0.8,0.1,0.1)	(0.5,0.2,0.3)	(0.6,0.3,0.1)	(0.7,0.1,0.1)
*A*_2_	(0.6,0.2,0.2)	(0.9,0,0.1)	(0.8,0.1,0)	(0.7,0.2,0.1)	(0.6,0.1,0.3)
*A*_3_	(0.7,0.1,0.2)	(0.7,0.2,0.1)	(0.8,0,0.2)	(0.7,0.1,0.2)	(0.6,0.1,0.2)
*A*_4_	(0.8,0.1,0.1)	(0.6,0.3,0.1)	(0.9,0.1,0)	(0.5,0.4,0.1)	(0.8,0.1,0.1)

In Phase II, the criteria weights are determined. First, decision makers reach a broad agreement that teaching contents (*C*_2_) should be first considered and finally the teaching link (*C*_4_) when assessing the teaching quality of a physical education college. Hence, they recognize the most important criterion *C*_2_ and the least important criterion *C*_4_, and repeat this process among the remaining criteria until all criteria are ranked in a descending order *C*_2_ ≻ *C*_1_ ≻ *C*_5_ ≻ *C*_3_ ≻ *C*_4_. Thereafter, experts evaluate the comparative importance degree between two adjacent criteria with PFNs, as shown in the second column of **Table 3**. For instance, if eight experts agree that teaching contents (*C*_2_) is more important than teaching attitude (*C*_1_) while the other two experts disagree, then the comparative importance degree *β*_2_ = (0.8, 0, 0.2).

**Table 3:** The weight of each criterion.

Criteria	Comparative importance degree *β*_*j*_	Comparative importance index *p*_(*j*)_	Importance degree *r*_(*j*)_	Weight *ω*_(*j*)_
*C*_2_	-	-	1	0.382
*C*_1_	(0.8,0,0.2)	0.6	0.625	0.239
*C*_5_	(0.6,0.2,0.2)	0.4	0.446	0.170
*C*_3_	(0.7,0.1,0.2)	0.5	0.297	0.114
*C*_4_	(0.5,0.2,0.3)	0.2	0.248	0.095

Then, using Eq (5), the comparative importance index of each criterion is calculated, as shown in the third columns of **Table 3**. For example, *p*_(*j*)_ = *S*(*β*_*j*_) ⇒ *p*_(2)_ = *S*(*β*_2_) = 0.8–0.2 = 0.6. By Eq (6), the importance degree of each criterion is computed, as shown in the fourth columns of **Table 3**. For instance, $r_{\left(j\right)}=\left\{\begin{array}{c} 1,\;j=1\\ r_{\left(j-1\right)}/(p_{\left(j\right)}+1),\;j=2,3,\ldots ,n \end{array}\right.\;\Rightarrow \;r_{\left(1\right)}=1$ and *r*_(2)_ = *r*_(1)_/(*p*_(2)_ + 1) = 1/(0.6 + 1) = 0.625. Last, the criteria weights are computed with Eq (7), as follows: $\omega_{\left(j\right)}=r_{\left(j\right)}/\sum_{j=1}^{n}r_{\left(j\right)}\;\Rightarrow \;\omega_{\left(1\right)}=r_{\left(1\right)}/\sum_{j=1}^{n}r_{\left(j\right)}=1/(1+0.625+0.446+0.297+0.248)=1/2.616\approx 0.382$, $\omega_{\left(2\right)}=r_{\left(2\right)}/\sum_{j=1}^{n}r_{\left(j\right)}=0.625/2.616\approx 0.239$, $\omega_{\left(3\right)}=r_{\left(3\right)}/\sum_{j=1}^{n}r_{\left(j\right)}=0.446/2.616\approx 0.170$, $\omega_{\left(4\right)}=r_{\left(4\right)}/\sum_{j=1}^{n}r_{\left(j\right)}=0.297/2.616\approx 0.114$ and $\omega_{\left(5\right)}=r_{\left(5\right)}/\sum_{j=1}^{n}r_{\left(j\right)}=0.248/2.616\approx 0.095$. That is, *ω*_1_ ≈ 0.239, *ω*_2_ ≈ 0.382, *ω*_3_ ≈ 0.114, *ω*_4_ ≈ 0.095 and *ω*_5_ ≈ 0.170.

In Phase III, the difference matrix is constructed. Because decision makers have no prior preference for these four colleges, their priority is equivalent, namely, $P_{A_{1}}=P_{A_{2}}=P_{A_{3}}=P_{A_{4}}=\frac{1}{4}$. As a result, a theoretical assessment matrix is built using Eq (9), as shown in **Table 4**. For example, $t_{11}=P_{A_{1}}\cdot \omega_{1}=\frac{1}{4}\times 0.239\approx 0.0598$.

**Table 4:** Theoretical assessment matrix *T*.

*T*	*ω*_1_	*ω*_2_	*ω*_3_	*ω*_4_	*ω*_5_
$P_{A_{1}}$	0.0598	0.0955	0.0285	0.0238	0.0425
$P_{A_{2}}$	0.0598	0.0955	0.0285	0.0238	0.0425
$P_{A_{3}}$	0.0598	0.0955	0.0285	0.0238	0.0425
$P_{A_{4}}$	0.0598	0.0955	0.0285	0.0238	0.0425

Since ${\tilde{\alpha }}_{1}^{-}=\min({\tilde{\alpha }}_{11},{\tilde{\alpha }}_{21},{\tilde{\alpha }}_{31},{\tilde{\alpha }}_{41})=(0.6,0.2,0.2)$, ${\tilde{\alpha }}_{2}^{-}=(0.6,0.3,0.1)$, ${\tilde{\alpha }}_{3}^{-}=(0.5,0.2,0.3)$, ${\tilde{\alpha }}_{4}^{-}=(0.5,0.4,0.1)$, ${\tilde{\alpha }}_{5}^{-}=(0.6,0.1,0.3)$, ${\tilde{\alpha }}_{1}^{+}=\max({\tilde{\alpha }}_{11},{\tilde{\alpha }}_{21},{\tilde{\alpha }}_{31},{\tilde{\alpha }}_{41})=(0.8,0.1,0.1)$, ${\tilde{\alpha }}_{2}^{+}=(0.9,0,0.1)$, ${\tilde{\alpha }}_{3}^{+}=(0.9,0.1,0)$, ${\tilde{\alpha }}_{4}^{+}=(0.7,0.2,0.1)$ and ${\tilde{\alpha }}_{5}^{+}=(0.8,0.1,0.1)$, then the distance between ${\tilde{\alpha }}_{j}^{+}$ and ${\tilde{\alpha }}_{j}^{-}$ can be computed according to Eq (3), as follows: $\begin{array}{l} d(\alpha_{1},\alpha_{2})=\sqrt{\left(|a_{1}-a_{2}{|}^{2}+|b_{1}-b_{2}{|}^{2}+|c_{1}-c_{2}{|}^{2}+|e_{1}-e_{2}{|}^{2}\right)}\\ \Rightarrow \;d({\tilde{\alpha }}_{1}^{+},{\tilde{\alpha }}_{1}^{-})=\sqrt{\left(|0.8-0.6{|}^{2}+|0.1-0.2{|}^{2}+|0.1-0.2{|}^{2}+|0-0{|}^{2}\right)}=\sqrt{0.06}\approx 0.2449 \end{array}$, $d({\tilde{\alpha }}_{2}^{+},{\tilde{\alpha }}_{2}^{-})=\sqrt{0.18}\approx 0.4243$, $d({\tilde{\alpha }}_{3}^{+},{\tilde{\alpha }}_{3}^{-})=\sqrt{0.26}\approx 0.5099$, $d({\tilde{\alpha }}_{4}^{+},{\tilde{\alpha }}_{4}^{-})=\sqrt{0.08}\approx 0.2828$ and $d({\tilde{\alpha }}_{5}^{+},{\tilde{\alpha }}_{5}^{-})=\sqrt{0.08}\approx 0.2828$. Furthermore, the distance ${\tilde{\alpha }}_{ij}$ and ${\tilde{\alpha }}_{j}^{-}$ can be calculated, such as $d({\tilde{\alpha }}_{11},{\tilde{\alpha }}_{1}^{-})=\sqrt{\left(|0.6-0.7{|}^{2}+|0.2-0.2{|}^{2}+|0.2-0.1{|}^{2}+|0-0{|}^{2}\right)}=\sqrt{0.02}\approx 0.1414$. Thereafter, a real assessment matrix is established using Eq (10), as shown in **Table 5**. For instance, $r_{ij}=t_{ij}\cdot \frac{d({\tilde{\alpha }}_{ij},{\tilde{\alpha }}_{j}^{-})}{d({\tilde{\alpha }}_{j}^{+},{\tilde{\alpha }}_{j}^{-})}\;\Rightarrow \;r_{11}=t_{11}\cdot \frac{d({\tilde{\alpha }}_{11},{\tilde{\alpha }}_{1}^{-})}{d({\tilde{\alpha }}_{1}^{+},{\tilde{\alpha }}_{1}^{-})}=0.0598\times \frac{0.1414}{0.2449}\approx 0.0345$.

**Table 5:** Real assessment matrix *R*.

*R*	*C*_1_	*C*_2_	*C*_3_	*C*_4_	*C*_5_
*A*_1_	0.0345	0.0637	0.0000	0.0119	0.0376
*A*_2_	0.0000	0.0955	0.0250	0.0238	0.0000
*A*_3_	0.0345	0.0318	0.0209	0.0315	0.0213
*A*_4_	0.0598	0.0000	0.0285	0.0000	0.0425

Based on Eq (11), a difference matrix is constructed in **Table 6**. For example, *g*_11_ = *t*_11_—*r*_11_ = 0.0598–0.0345 = 0.0253.

**Table 6:** Difference matrix *G*.

*G*	*C*_1_	*C*_2_	*C*_3_	*C*_4_	*C*_5_
*A*_1_	0.0253	0.0318	0.0285	0.0119	0.0049
*A*_2_	0.0598	0.0000	0.0035	0.0000	0.0425
*A*_3_	0.0253	0.0637	0.0076	-0.0077	0.0213
*A*_4_	0.0000	0.0955	0.0000	0.0238	0.0000

In Phase IV, the ranking orders are acquired. First, let ∇_*j*_ = 0.01, Δ_*j*_ = 0.02 and Λ_*j*_ = 0.05, then the concordance degree between two physical education colleges is computed using Eq (12), as shown in **Table 7**. For instance, $\begin{array}{l} CD(A_{i},A_{k})=\sum_{j=1}^{m}\left(\omega_{j}\cdot \Psi (g_{ij},g_{kj})\right)\\ \Rightarrow \;CD(A_{1},A_{2})=\sum_{j=1}^{5}\left(\omega_{j}\cdot \Psi (g_{1j},g_{2j})\right)=0.239\times 1+0.382\times 0+0.114\times 0+0.095\times 0.81+0.170\times 1=0.48595\approx 0.4860 \end{array}$.

**Table 7:** Concordance degree *CD*(*A*_*i*_, *A*_*k*_).

*CD*(*A*_*i*_, *A*_*k*_)	*A*_1_	*A*_2_	*A*_3_	*A*_4_
*A*_1_	1.0000	0.4860	0.7948	0.6470
*A*_2_	0.5910	1.0000	0.5910	0.5910
*A*_3_	0.5092	0.6180	1.0000	0.5910
*A*_4_	0.6000	0.5230	0.5230	1.0000

Thereafter, based on Eq (13), their credibility degree is calculated in **Table 8**. For example, $CI(A_{i},A_{k})=CD(A_{i},A_{k})\cdot \prod_{j=1}^{m}DI_{j}(A_{i},A_{k})\;\Rightarrow \;CI(A_{1},A_{2})=CD(A_{1},A_{2})\cdot \prod_{j=1}^{5}DI_{j}(A_{1},A_{2})=0.4860\times 1\times 1\times 1\times 1\times 1=0.4860$.

**Table 8:** Credibility degree *CI*(*A*_*i*_, *A*_*k*_).

*CI*(*A*_*i*_, *A*_*k*_)	*A*_1_	*A*_2_	*A*_3_	*A*_4_
*A*_1_	1.0000	0.4860	0.7948	0.6470
*A*_2_	0.5910	1.0000	0.5910	0.0000
*A*_3_	0.5092	0.0000	1.0000	0.5910
*A*_4_	0.0000	0.0000	0.5230	1.0000

Last, the ranking index of each physical education college is obtained with Eq (14), as follows: $\begin{array}{l} RI(A_{i})=\sum_{k=1}^{n}CI(A_{i},A_{k})-\sum_{k=1}^{n}CI(A_{k},A_{i})\\ \Rightarrow \;RI(A_{1})=\sum_{k=1}^{4}CI(A_{1},A_{k})-\sum_{k=1}^{4}CI(A_{k},A_{1})=(1+0.4860+0.7948+0.6470)-(1+0.5910+0.5092+0)=0.8276\approx 0.828, \end{array}$ *RI*(*A*_2_) ≈ 0.696, *RI*(*A*_3_) ≈ -0.809 and *RI*(*A*_4_) ≈ -0.715. Since *RI*(*A*_1_) > *RI*(*A*_2_) > *RI*(*A*_4_) > *RI*(*A*_3_), the final ranking order is *A*_1_ ≻ *A*_2_ ≻ *A*_4_ ≻ *A*_3_, and the best physical education college is *A*_1_.

## Analyses and discussions

In this section, analyses and discussions are made to verify the effectiveness of our method.

### Sensitivity analyses

To testify the sensitivity of the proposed method, the variations of ranking results are analyzed by changing the criteria weights in Section 4. Assume an objective criteria weight vector is *w*^*o*^ = (0.200,0.200,0.200,0.200,0.200), then the comprehensive weight vector is updated as *w* = *ζ*⋅*w*^*o*^ + (1 - *ζ*)⋅ω, where *ζ* ∈ [0,1] is the weight coefficient and *ω* = (0.239,0.382,0.114,0.095,0.170). The ranking orders with different values of *ζ* are listed in **Table 9**.

**Table 9:** Ranking orders with different *ζ* values.

*ζ* value	Weight vector	Ranking index	Ranking order	Best college	*ƛ* value	ℏ value
*ζ* = 0	(0.239,0.382, 0.114,0.095, 0.170)	*RI*(*A*_1_) ≈ 0.828, *RI*(*A*_2_) ≈ 0.696, *RI*(*A*_3_) ≈ -0.809, *RI*(*A*_4_) ≈ -0.715.	*A*_1_ ≻ *A*_2_ ≻ *A*_4_ ≻ *A*_3_	*A*_1_	-	-
*ζ* = 0.1	(0.235,0.364, 0.123,0.105, 0.173)	*RI*(*A*_1_) ≈ 0.806, *RI*(*A*_2_) ≈ 0.679, *RI*(*A*_3_) ≈ -0.781, *RI*(*A*_4_) ≈ -0.703.	*A*_1_ ≻ *A*_2_ ≻ *A*_4_ ≻ *A*_3_	*A*_1_	1.0	1.732
*ζ* = 0.2	(0.231,0.346, 0.131,0.116, 0.176)	*RI*(*A*_1_) ≈ 0.790, *RI*(*A*_2_) ≈ 0.661, *RI*(*A*_3_) ≈ -0.671, *RI*(*A*_4_) ≈ -0.781.	*A*_1_ ≻ *A*_2_ ≻ *A*_3_ ≻ *A*_4_	*A*_1_	0.8	1.386
*ζ* = 0.3	(0.227,0.327, 0.140,0.127, 0.179)	*RI*(*A*_1_) ≈ 0.774, *RI*(*A*_2_) ≈ 0.639, *RI*(*A*_3_) ≈ -0.515, *RI*(*A*_4_) ≈ -0.898.	*A*_1_ ≻ *A*_2_ ≻ *A*_3_ ≻ *A*_4_	*A*_1_	1.0	1.732
*ζ* = 0.4	(0.223,0.309, 0.149,0.137, 0.182)	*RI*(*A*_1_) ≈ 0.752, *RI*(*A*_2_) ≈ 0.615, *RI*(*A*_3_) ≈ -0.335, *RI*(*A*_4_) ≈ -1.033.	*A*_1_ ≻ *A*_2_ ≻ *A*_3_ ≻ *A*_4_	*A*_1_	1.0	1.732
*ζ* = 0.5	(0.220,0.291, 0.157,0.147, 0.185)	*RI*(*A*_1_) ≈ 0.590, *RI*(*A*_2_) ≈ 0.504, *RI*(*A*_3_) ≈ -0.037, *RI*(*A*_4_) ≈ -1.057.	*A*_1_ ≻ *A*_2_ ≻ *A*_3_ ≻ *A*_4_	*A*_1_	1.0	1.732
*ζ* = 0.6	(0.216,0.273, 0.165,0.158, 0.188)	*RI*(*A*_1_) ≈ 0.260, *RI*(*A*_2_) ≈ 0.257, *RI*(*A*_3_) ≈ -0.327, *RI*(*A*_4_) ≈ -0.843.	*A*_3_ ≻ *A*_1_ ≻ *A*_2_ ≻ *A*_4_	*A*_3_	0.4	0.693
*ζ* = 0.7	(0.212,0.255, 0.174,0.168, 0.191)	*RI*(*A*_1_) ≈ -0.050, *RI*(*A*_2_) ≈ -0.084, *RI*(*A*_3_) ≈ 0.701, *RI*(*A*_4_) ≈ -0.568.	*A*_3_ ≻ *A*_1_ ≻ *A*_2_ ≻ *A*_4_	*A*_3_	1.0	1.732
*ζ* = 0.8	(0.208,0.236, 0.183,0.179, 0.194)	*RI*(*A*_1_) ≈ -0.363, *RI*(*A*_2_) ≈ -0.123, *RI*(*A*_3_) ≈ 0.769, *RI*(*A*_4_) ≈ -0.283.	*A*_3_ ≻ *A*_2_ ≻ *A*_4_ ≻ *A*_1_	*A*_3_	-0.4	-0.693
*ζ* = 0.9	(0.204,0.218, 0.191,0.190, 0.197)	*RI*(*A*_1_) ≈ -0.644, *RI*(*A*_2_) ≈ -0.175, *RI*(*A*_3_) ≈ 0.881, *RI*(*A*_4_) ≈ -0.063.	*A*_3_ ≻ *A*_4_ ≻ *A*_2_ ≻ *A*_1_	*A*_3_	0.2	0.346
*ζ* = 1.0	(0.200,0.200, 0.200,0.200, 0.200)	*RI*(*A*_1_) ≈ -0.957, *RI*(*A*_2_) ≈ -0.211, *RI*(*A*_3_) ≈ 1.102, *RI*(*A*_4_) ≈ 0.066.	*A*_3_ ≻ *A*_4_ ≻ *A*_2_ ≻ *A*_1_	*A*_3_	1.0	1.732

Toss explore the relationship between ranking orders under different *ζ* valuesss, the Spearman’s rank-correlation test [37] is adopted with the following two parameters:

$$ƛ=1-\frac{6\cdot \sum_{i=1}^{m}{\left(dis(A_{i})\right)}^{2}}{m(m^{2}-1)},$$ (15)

$$\hbar =ƛ\cdot \sqrt{\left(m-1\right)},$$ (16)

where ƛ ∈ [-1,1], *m* is the number of alternatives and *dis*(*A*_*i*_) is the difference degree of alternative *A*_*i*_ under different ranking results.

When the value of ƛ is close to 1 (or -1), it means a close correlation between two rankings. Thus, based on Eqs (15)–(16), the ƛ and ℏ values are computed, as shown in the sixth and seventh columns of **Table 9**. For instance, when the *ζ* value varies from 0.1 to 0.2, the ranking order changes from *A*_1_ ≻ *A*_2_ ≻ *A*_4_ ≻ *A*_3_ to *A*_1_ ≻ *A*_2_ ≻ *A*_3_ ≻ *A*_4_, then using Eq (15), $ƛ=1-\frac{6\cdot \sum_{i=1}^{m}{\left(dis(A_{i})\right)}^{2}}{m(m^{2}-1)}=1-\frac{6\times (0^{2}+0^{2}+1^{2}+1^{2})}{4\times (4^{2}-1)}=0.8$, and using Eq (16), $\hbar =ƛ\cdot \sqrt{\left(m-1\right)}=0.8\times \sqrt{3}\approx 1.386$.

From **Table 9**, it can be seen that the best college *A*_1_ is recognized when 0 ≤ *ζ* < 0.6, while the ranking orders change a lot when *ζ* value varies from 0.5 to 0.6. The reason may be that with the increase of *ζ* value, the significance of teaching contents *C*_2_ and teaching attitude *C*_1_ is diminished. At the same time, with the increase of weights of other criteria (teaching approaches *C*_3_, teaching effect *C*_4_ and teaching link *C*_5_), the ranking orders are dissimilar with different *ζ* values (*ζ* ≥ 0.6). On the contrary, when the importance of teaching contents *C*_2_ and teaching attitude *C*_1_is emphasized, the ranking orders keep relatively stable and college *A*_1_ is highlighted.

### Comparison analyses

Several different decision-making approaches are applied to deal with the teaching quality evaluation of physical education.

1. Approach 1: This approach is presented by Wei [12]. He defined the weighted arithmetic average aggregation operator of PFNs and then proposed Approach 1 on the basis of this operator.
2. Approach 2: This approach is based on the weighted geometric average aggregation operator of PFNs [12].
3. Approach 3: This approach is proposed by Wang et al. [19]. They defined the distance of PFNs, and then extended the classical MABAC model with picture fuzzy information.
4. Approach 4: This approach is a modified WDBA method in picture fuzzy environments [22].
5. Approach 5: This approach is introduced by Liang et al. [18]. They combined EDAS with ELECTRE models to get the ranking orders of alternatives.
6. Approach 6: This approach is a classical MAIRCA approach, whose inputs are PFNs. The discrepancy between Approach 6 and our approach is the determination of ranking index of physical education colleges. That is, the ranking index of physical education colleges is computed by $\sum_{j=1}^{n}g_{ij}$in Approach 6. The smaller the value of $\sum_{j=1}^{n}g_{ij}$, the better the physical education college *A*_*iss*_.

Then, the ranking orders using the above six approaches are obtained and listed in **Table 10**.

**Table 10:** Ranking orders with different approaches.

Approach	Ranking order	Best college	Worst college	Total gap *TG*
Approach 1 [12]	*A*_4_ ≻ *A*_1_ ≻ *A*_2_ ≻ *A*_3_	*A*_4_	*A*_3_	4.00
Approach 2 [12]	*A*_2_ ≻ *A*_3_ ≻ *A*_4_ ≻ *A*_1_	*A*_2_	*A*_1_	2.17
Approach 3 [19]	*A*_4_ ≻ *A*_1_ ≻ *A*_2_ ≻ *A*_3_	*A*_4_	*A*_3_	4.00
Approach 4 [22]	*A*_2_ ≻ *A*_1_ ≻ *A*_4_ ≻ *A*_3_	*A*_2_	*A*_3_	1.50
Approach 5 [18]	*A*_1_ ≻ *A*_3_ ≻ *A*_2_ ≻ *A*_4_	*A*_1_	*A*_4_	1.33
Approach 6	*A*_1_ ≻ *A*_2_ ≻ *A*_3_ ≻ *A*_4_	*A*_1_	*A*_4_	0.83
MAIRCA-ELECTRE	*A*_1_ ≻ *A*_2_ ≻ *A*_4_ ≻ *A*_3_	*A*_1_	*A*_3_	0.00

From **Table 10**, it can be seen that diverse ranking results are obtained with dissimilar approaches. To determine the optimal ranking order, a scoring mechanism is employed. That is, a higher ranking score is assigned to a better alternative. Take the ranking order *A*_4_ ≻ *A*_1_ ≻ *A*_2_ ≻ *A*_3_ obtained by Approach 1 as an example, the ranking score of alternative *A*_4_ is *RS*_1_(*A*_4_), that of *A*_1_ is *RS*_1_(*A*_1_) = 3, that of *A*_2_ is *RS*_1_(*A*_2_) = 2, and that of *A*_3_ is *RS*_1_(*A*_3_) = 1. In this manner, the ranking orders with above six approaches and our method are scored in turn. As a result, the total ranking score of each alternative is computed by summation as follows: *RS*(*A*_1_) = 3 + 1 + 3 + 3 + 4 + 4 + 4 = 22, *RS*(*A*_2_) = 20, *RS*(*A*_3_) = 12 and *RS*(*A*_4_) = 16. Because *RS*(*A*_1_) > *RS*(*A*_2_) > *RS*(*A*_4_) > *RS*(*A*_3_), the optimal ranking order is *A*_1_ ≻ *A*_2_ ≻ *A*_4_ ≻ *A*_3_. It is clear that the ranking order with MAIRCA-ELECTRE approach is the same with the optimal ranking order. It demonstrates that our approach is more pertinent than other six approaches in disposing physical education teaching quality evaluation issues.

Then, the method proposed in [38] is adopted to measure the gap between each ranking order listed in **Table 10** and the optimal ranking order. That is, their gap can be determined with the following equation:

$$TG=\sum_{i=1}^{m}\left|\frac{h_{i}-H_{i}}{H_{i}}\right|,$$ (17)

where *H*_*i*_ is the optimal ranking order of alternative *A*_*i*_, and *h*_*i*_ is the ranking order of alternative *A*_*i*_ with an approach listed in **Table 10**.

Based on Eq (15), the total gap between the results of each approach and the optimal ranking order is calculated, as shown in the last column of **Table 10**. It is true that Approach 1 has the largest gap, followed by Approach 2. Both the gap of method 5 and the gap of method 4 are smaller than that of Approach 3. Furthermore, our approach (MAIRCA-ELECTRE) achieves the smallest gap, followed by Approach 6. Possible reasons for their differences are: Approach 1, 2, 3, 4 and 6 cannot deal with the situation where evaluation criteria are not compensatory. Additionally, Approach 1 and 2 are based on different aggregation operators of PFNs. In this case, some evaluation information may be lost or distorted during the aggregation process. Although Approach 5 can tackle non-compensatory criteria, its average solutions are calculated using aggregation operators in the difference matrix construction process with the EDAS method. In this case, it may not avoid the information loss or distortion problem. Overall, results show that the proposed MAIRCA-ELECTRE approach is feasible and the most appropriate among these approaches.

## Discussions

The proposed approach combines the MAIRCA method for establishing the difference matrix, and the ELECTRE method for getting the ranking result of physical education colleges. The largest advantages of our method are two-fold. First, compared with other popular methods (such as VIKOR, MARCOS [39], DEMATEL (Decision Making Trial and Evaluation Laboratory) and FUCOM (Full Consistency Method)), the distance-based MAIRCA method is easily implemented and can reduce information loss as much as possible. On the other hand, compared with some classical approaches (such as the TOPSIS, WDBA and MABAC), the ELECTRE method can effectively handle evaluation criteria with non-compensate. Comparative analyses reveal that our approach is more suitable in settling decision-making problems with non-compensatory criteria. Furthermore, SWARA is introduced for recognizing criteria relative significance and weights subjectively [40]. Compared with other weight-calculation technologies (such as AHP and BWM (Best-Worst method)), it gives the chance for experts or decision makers to determine their priority according to the current conditions of social and economy [41]. One limitation of the model may be that all decision makers are assumed to have complete rationality and equal weights, which should be overcome by introducing other theories in the future.

## Conclusions

Physical education is very important in promoting comprehensive development of students and cultivating sports specialists. This study focused on the teaching quality evaluation of physical education with a novel fuzzy MCDM support framework. First, the teaching quality evaluation indexes of physical education were identified. With respect to the intricacy of teaching quality evaluation and the diversity of human beings’ opinions, PFNs were used to indicate fuzzy decision making data with four membership functions. Then, the modified SWARA model was established to determine the weight vector of evaluation criteria in picture fuzzy environments. Thereafter, the MAIRCA approach was extended with PFNs to construct the difference matrix. Furthermore, the ELECTRE III method is utilized to get the ranking orders of physical education colleges. The main advantage of such approach is that it can properly deal with non-compensatory criteria during the teaching quality evaluation process. Comparative analyses indicated that the proposed approach was workable and beneficial for the teaching quality evaluation of physical education, and could offer guidance for the performance appraisal and selection of physical education teachers.

However, there are still some limitations of the proposed methodology. For example, experts are assumed to have equal weights, which may be not appropriate in some cases. In the future, some weight-calculation technologies should be explored to determine the weight of each decision maker especially in a group decision-making environment. Second, evaluators are regarded as completely rational. In the future, the proposed approach can be improved by considering the limited rationality or psychological characteristics of decision makers during the evaluation process.
